This article has been retracted.

# Analysis on the Social Environment of College Students' Rural Employment and Entrepreneurship

**DOI:** 10.1155/2022/3475897

**Published:** 2022-07-12

**Authors:** Wenguo Chai

**Affiliations:** Xinyang Vocational and Technical College, Xinyang 464000, China

## Abstract

This paper aims to further solve the risks encountered by college students in the process of employment and entrepreneurship in rural areas and improve the success rate of employment and entrepreneurship. It presents a method of social environment analysis based on college students' rural employment and entrepreneurship. This method deeply understands the employment and entrepreneurship environment of college students, deeply analyzes and identifies the constituent elements of college students' rural employment and entrepreneurship environment, and takes the social environment of college students' rural employment and entrepreneurship as the research object. With the help of questionnaire survey and data analysis, the survey shows that, in the channel selection of job hunting in the future, up to 77.20% choose to apply for a job through job fairs, and 69.60% will use advertising media such as networks and newspapers; 26.50% will apply for jobs through the talent market; 31.30% will apply for a job through relatives and friends; 15.40% will apply for jobs through independent entrepreneurship. This paper constructs the evaluation model of entrepreneurship and employment environment from the perspective of subjectivity and puts forward the optimization strategy of entrepreneurship and employment environment from four fields: policy environment, capital environment, education environment, and cultural environment.

## 1. Introduction

Since the beginning of the new century, with China's accession to the World Trade Organization and the deepening of reform and opening up, China's industrial economy has developed very well. At the same time, the industrial scale has been continuously expanded and China's economic structure has been gradually improved. It can be said that the market economy under the socialist system with Chinese characteristics has undergone earth-shaking changes under the trend of stable growth [1]. The employment and entrepreneurship environment has also changed greatly. Taking entrepreneurship as an example, at this stage, various entrepreneurial groups in China emerge one after another. In this process, private enterprises and a large number of small and medium-sized enterprises have developed rapidly, and the number of employees in private enterprises is also increasing year by year. Since China put forward the Rural Revitalization Strategy, the vast rural areas have provided a good platform for the employment and Entrepreneurship of college students, and the employment and entrepreneurship experience of college students in rural areas has also injected more fresh blood into the development of rural areas and the implementation of rural strategy. Nowadays, the problem of employment and entrepreneurship environment in rural areas is the result of the interaction of many factors, and it is also the concentrated embodiment of many problems. A good employment and entrepreneurship environment plays a vital role for college students to take root in rural areas [2]. Therefore, this study aims to gradually improve the employment and entrepreneurship environment in rural areas and create more powerful conditions for college students to take root in rural areas. See Figure 1.

## 2. Literature Review

V Bhatt and others found that there are numerous scholars studying the employment of college students in China, and a hundred schools of thought contend [3]. Mert and others took a university as an example to study the employment of college students from the perspective of social capital [4]. Chatzichristos and others took social capital as the starting point and considered the difficult employment of College Students under the background of segmented labor market and fragmented social security [5]. Gardaevi and others analyzed the current situation, characteristics, and socioeconomic impact of college students' employment from the perspective of human capital theory and made a specific analysis of Chinese college students' employment from the perspective of supply and demand on the basis of the previously mentioned theory [6]. Based on the case investigation and access to relevant materials, by introducing the western labor market division theory and combined with the current development of China's labor market, Veselov and others put forward the application of a new theory—“three-level and five-tier” labor market division theory—to study the employment problem of college students in China, so as to provide a new idea for solving the employment problem of college students [7]. Finally, Golsifid-Alavi and others put forward countermeasures and suggestions to solve the employment problem of college students from this new perspective [8]. Adedoyin and others used the sampling survey method to select six representative college graduates for follow-up survey and conducted in-depth analysis and research on the social support network in college students' employment by using the theories of social support network and social resources [9]. Moriggi and others revealed the internal characteristics of the social support network for college students' employment by analyzing the impact and supporting role of the social support network for college students' employment. Through the understanding and analysis of these characteristics, they put forward constructive countermeasures on how to use these characteristics and influencing factors to solve the employment problem of college students. However, scholars or monographs who have conducted special research on the employment situation of this special group of returned rural college students have not found that only some media have a simple description of some return employment policies [10].

Obschonka and others found that western developed countries have also experienced or are experiencing the social problems of high unemployment rate of college students in the stage of popularization and popularization of higher education. All countries have made a series of fruitful explorations [11]. For example, all walks of life in the UK have suffered from the financial crisis. The first thing to bear the brunt is the employment of British college graduates. In view of the severe employment situation of college graduates, the British government has launched various measures to solve the difficult employment problem of college students. The first is the “national internship plan.” The British government has asked public institutions, charities, and economic departments to absorb a certain number of college graduates for internships. Interns can not only get a certain income but also take this opportunity to accumulate work experience and lay the foundation for ideal employment in the future. All major enterprises have responded positively to the government's call. Huang found that compared with western countries, although China has differences in political system and degree of marketization, the experience and lessons of these countries are still worthy of our reference [12]. The construction of social support network for the group employment of rural returned college students can also draw nutrition from it and gradually build and improve it. Western scientists have conducted a lot of in-depth and meticulous research on the business environment through scientific research outside China, forming a mature theoretical program. Chinese scholars have also carried out some theoretical research and applied science from the research of foreign research combined with the actual situation in China. Overall, the existing business environment research has matured, but the number of research papers on the “student” industry environment is limited; the research content is not deep enough. The research focus is mainly on the integration of college students' entrepreneurial environment, the analysis of current situation, and countermeasures and suggestions, while the research on college students' entrepreneurial environment is still relatively limited. There is not enough research. The research process is usually based on quality and data analysis, although some studies use the process to assess the student business environment. The research level is not high enough, and major newspapers and magazines have also published some statements about the business environment. Therefore, it is necessary to further strengthen the research on the business environment of students.

## 3. Evaluation of College Students' Employment and Entrepreneurship Environment

### 3.1. Evaluation Method

#### 3.1.1. Factor Analysis

Factor analysis is one of the commonly used dimensionality reduction analysis methods in multivariate statistics. It describes the relationship between index variables by constructing some unobservable random variables, to achieve the purpose of dimensionality reduction, simplification, and comprehensive evaluation. There are two types of analysis: *R*-type factor analysis and *Q*-type factor analysis. In this paper, *R*-type analysis is selected as the main analysis method. Its mathematical model is as follows:

(1) $$\begin{array}{c} \left\{\begin{array}{c} X_{1}=a_{11}F_{1}+a_{12}F_{2}+,\text{…},a_{1m}F_{m}+\varepsilon_{1},\\ X_{2}=a_{21}F_{1}+a_{22}F_{2}+,\text{…},a_{2m}F_{m}+\varepsilon_{2},\\ ......,\\ X_{p}=a_{p1}F_{1}+a_{p2}F_{2}+,\text{…},a_{pm}F_{m}+\varepsilon_{3}. \end{array}\right) \end{array}$$

And the previously mentioned formula meets

(2) $$\begin{array}{c} \left(i\right)m\leq p,\\ \left(ii\right)Cov\left(F,\varepsilon \right)=0. \end{array}$$

In the previously mentioned formula, *F* and *ε* are irrelevant.

(3) $$\begin{array}{c} \left(iii\right)D\left(F\right)=\left[\begin{array}{cc} 1 & 0\\ 0 & 1 \end{array}\right]=I_{m}. \end{array}$$

That is, formula *F*_1_…*F*_*m*_ is irrelevant and the variance is 1.

(4) $$\begin{array}{c} \begin{array}{cc} \; & D\left(\varepsilon \right) \end{array}=\left[\begin{array}{ccc} \delta_{1}^{2} & \; & 0\\ \; & \delta_{2}^{2} & \;\\ 0 & \; & \delta_{p}^{2} \end{array}\right]. \end{array}$$

That is, formula *ε*_1_...*ε*_*m*_ is irrelevant and the variance is different, of which

(5) $$\begin{array}{c} X={\left(X_{1},\text{…},X_{p}\right)}^{\prime }. \end{array}$$

The previously mentioned formula is a *p*-dimensional random vector composed of *P* indexes directly obtained through observation.

(6) $$\begin{array}{c} F={\left(F_{1},\text{…},F_{m}\right)}^{\prime }. \end{array}$$

The previously mentioned formula is the unobservable vector (the common factor extracted by factor analysis). *a*_*ij*_ is called factor load, that is, the load of the *i*-th variable on the *j*-th common factor; *ε* is a special factor of *X*, and the covariance matrix of *ε* is a diagonal matrix in theory [13].

#### 3.1.2. Factor Score and Its Application

It best describes the relationship between the original variables. Using the best possible representation of the old variable will help explain the characteristics of the study material. Therefore, it is necessary to express the common factor as a linear combination of variables; that is,

(7) $$\begin{array}{c} F_{j}=\beta_{j1}X_{1}+\text{…}+\beta_{jp}X_{p},\;j=1,\text{…},p. \end{array}$$

The previously mentioned models are job scores that can be used to calculate the score for each model.

The mathematical model of factor analysis is a linear combination of variables expressed as common factors:

(8) $$\begin{array}{c} X_{i}=a_{i1}F_{1}+\text{…}+ai_{m}F_{m},\;i=1,\text{…},p. \end{array}$$

According to the factor score, each factor can be sorted to find out the key factors, and then targeted management measures can be put forward.

#### 3.1.3. Calculation Steps of Factor Analysis Method

Take the following original data as an example to illustrate the calculation steps of factor analysis method as shown in Table 1.

(1) Standardize the original data and record it as *x*_*ij*_
(2) Establish the correlation coefficient matrix of variables as follows:
  (9) $$\begin{array}{c} R={\left(r_{ij}\right)}_{p\times p}, \end{array}$$
where
  (10) $$\begin{array}{c} r_{ij}=\frac{\sum_{a=1}^{n}\left(x_{ai}-\bar{x_{i}}\right)\left(x_{aj}-\bar{x_{j}}\right)}{\sqrt{\sum_{a=1}^{n}{\left(x_{ai}-\bar{x_{i}}\right)}^{2}}•\sqrt{\sum_{a=1}^{n}{\left(x_{aj}-\bar{x_{j}}\right)}^{2}}}. \end{array}$$
This leads to
  (11) $$\begin{array}{c} r_{ij}=\frac{1}{n}\sum_{a=1}^{n}x_{ai}•x_{aj}. \end{array}$$
(3) The eigenvalue of *R* and the corresponding unit eigenvector are obtained and recorded as
  (12) $$\begin{array}{c} \lambda_{1}\geq \lambda_{2}\geq \text{…}\geq \lambda_{p}>0,\\ u_{1},u_{2},\text{…},u_{p},\\ U=\left(u_{1},u_{2},\text{…},u_{p}\right)=\left[\begin{array}{cccc} u_{11} & u_{12} & ... & u_{1p}\\ u_{21} & u_{22} & ... & u_{2p}\\ ... & ... & ... & ...\\ u_{p1} & u_{p2} & ... & u_{pp} \end{array}\right]. \end{array}$$
According to the ratio of cumulative contribution rate,
  (13) $$\begin{array}{c} \frac{\sum_{i=1}^{m}\lambda_{i}}{\sum_{i=1}^{p}\lambda_{i}}. \end{array}$$
Take the first *m* eigenvalues (eigenvalues greater than 1 in practical operation) and the corresponding eigenvectors to write the factor load matrix:
  (14) $$\begin{array}{c} A=\left[\begin{array}{cccc} a_{11} & a_{12} & ... & a_{1m}\\ a_{21} & a_{22} & ... & a_{2m}\\ ... & ... & ... & ...\\ a_{p1} & a_{p2} & ... & a_{pm} \end{array}\right]=\left[\begin{array}{cccc} u_{11}\sqrt{\lambda_{1}} & u_{12}\sqrt{\lambda_{2}} & ... & u_{1m}\sqrt{\lambda_{m}}\\ u_{21}\sqrt{\lambda_{1}} & u_{22}\sqrt{\lambda_{2}} & ... & u_{2m}\sqrt{\lambda_{m}}\\ ... & ... & ... & ...\\ u_{p1}\sqrt{\lambda_{1}} & u_{p2}\sqrt{\lambda_{2}} & ... & u_{11}\sqrt{\lambda_{m}} \end{array}\right]. \end{array}$$
(4) Perform maximum variance orthogonal rotation on a.
(5) The scores of each factor are calculated and sorted. Finally, the influence degree of different factors on events is determined according to the different factor scores [14].

### 3.2. Structural Equation Model

Equivalent models usually consist of measurement models and structural models. Measurement models are used to influence the relationship between latent variables and clinical indicators. Structural model is a model used to show the relationship between potential variables and potential variables. In the study of structural equation model, we call the phenomenon that cannot be measured directly as latent variable. Variables that can be measured directly are called observation variables.

The construction of structural equation model mainly includes the following four steps.

1. *Model Construction.* According to the theory and previous relevant research results, a theoretical model is constructed, and then, the relationship between variables is studied and analyzed by using structural equation model [15]. The contents of model construction include the relationship between observation variables and latent variables and the relationship between the latent variables.
2. *Model Estimation.* Generally, generalized multiplication or maximum likelihood method is used to estimate the model parameters. Among them, the most efficient method is the most widely used method.
3. *Model Evaluation.* After the construction of the model, the evaluation is carried out, including the appropriateness analysis of the solution of the structural equation and the rationality analysis of the relationship between model parameters and preset models. The fitting relationship is evaluated and compared with the fitting index of the alternative model.
4. *Model Modification.* If the model has not been well fitted, it is necessary to modify and reset the model. In this case, it is necessary to modify, delete, or add model parameters [16]. The fitting degree of the model can be increased by resetting the parameters.

## 4. Investigation on College Students' Employment and Entrepreneurship Intention

### 4.1. Purpose and Significance of Investigation

Based on the previous analysis of the current employment situation of college students in Xinjiang, this chapter investigates and analyzes the sample of an agricultural university in the form of questionnaire and analyzes the choice of rural employment intention of agricultural college students based on the survey data. According to the analysis of the current employment mode, characteristics, and employment situation of college students in an agricultural university, we can objectively grasp the current employment situation of college students in an agricultural university and also provide a reference basis for the construction and evaluation of subsequent theoretical models [17].

### 4.2. Basic Information of Investigation

#### 4.2.1. Questionnaire Distribution

The questions designed in the questionnaire involve the respondents' gender, nationality, major, registered residence location, and other contents related to “college Students' employment intention.” Four hundred questionnaires were distributed, and 391 questionnaires were recovered, with a recovery rate of 97.75%. Among them, there were 360 valid questionnaires, and the effective questionnaire rate was 90.00%. Among the respondents, the proportion of men is 56.00% and that of women is 44.00%, which tends to be balanced and meets the requirements of effective sample investigation [18].

#### 4.2.2. Analysis of Basic Information of Respondents

The survey found that most of the students of an agricultural university come from Rural Youth League farms, but their employment intention focuses on large and medium-sized cities. In an agricultural college, most of the nrolment sources are rural areas and regimental areas, and most of the training categories are majors in agriculture, forestry, animal husbandry, and fishery. The result of the survey is that nearly 50% of the students come from rural areas, towns, and league farms and 32% from small and medium-sized cities. 27% of the students are willing to work in the political centers of various prefectures, and 9% of the students hope to develop outside Xinjiang. Only 12% of students are willing to return to the county or rural areas to work. See Figures 2 and 3.

Through the survey, it is found that the amount of students' daily living expenses is divided into several levels (see Figure 4). The proportion of living expenses below 200 yuan per month is zero, which is also in line with the current consumption level of a university [19]. Among them, the monthly living expenditure is 400–1000 yuan, accounting for 76%, which is the main level area of students' consumption expenditure at present. On the one hand, the amount of student consumption expenditure is high, but on the other hand, its economic source is very single (see Figure 5). Among them, 74% of the students currently rely on external economic sources, including 58% from home, 15% from schools, and 0.7% from social assistance. The rest of the students who supplement their financial resources by doing part-time jobs account for 20%.

Through the survey, the graduates of an agricultural college have a strong sense of employment pressure, especially the majors related to agriculture, and often encounter neglect when applying for a job. The job hunting season in 2021 has come, and the graduating students are making a lot of preparations for entering the society, accompanied by a strong sense of employment pressure [20]. Therefore, a comprehensive understanding of employment pressure and reasonable response and release is very important. According to the survey, the sources of employment pressure of students are mainly from four aspects: personal pressure, school pressure, family pressure, and social pressure. From low to high, school pressure accounts for 11%, social pressure 19%, family pressure 31%, and personal pressure 39% (see Figure 6). This shows that, at present, the source of students' employment pressure mainly lies in themselves and their families. Considering personal feelings and family hopes, students should not only meet their own needs but also satisfy their families.

### 4.3. Analysis of Employment Survey Results

#### 4.3.1. Analysis of Employment Situation

Of the 360 university graduate students, only 8% thought the current situation was good and easy, 31% thought the current situation was good, and about 61% thought the current situation was difficult and difficult [21]. To a certain extent, this means that college students still lack of confidence and self-confidence when they first step into the workplace. At the same time, it also explains the psychological state of the talent market for talent supply (see Figure 7).

In the survey, up to 77.00% of college students believe that China's development and college students' employment trend will recover slowly in the next few years, 15.40% of college students believe that China's economic development and college students' employment trend will be in a downturn in the next few years, and the rest believe that the situation is relatively stable and has little fluctuation (see Figure 8).

The survey shows that 53.80% of college students believed that they need to improve their quality and accumulate relevant work or internship experience; 46.00% believed that professional knowledge and skills needed to be improved; 38.50% of them believed that they needed to improve their ability to withstand pressure and overcome difficulties; 42.00% of them believed that communication and coordination skills and basic problem-solving skills needed to be improved (see Figure 9).

To sum up, from the perspective of the employment situation, college students generally feel that the employment pressure is still quite large. However, in order to improve their own quality, they expect to show their skills when the employment situation is getting better in the future, accumulate and wait, adapt and introvert at the same time, and do not waste time, but complain more [22].

#### 4.3.2. Employment Tendency Analysis

The survey found that the proportion of college Students' employment intention inclined to administrative institutions, state-owned enterprises, joint ventures, scientific research institutes, military, and independent entrepreneurship is 61.40%, 53.70%, 23.60%, 15.40%, 36.30%, and 7.70% (see Figure 10).

It is found in the survey that 64.30% choose cities and 21.40% choose rural areas. The rest think it depends on the situation and is uncertain (see Figure 11) [23]. 21.40% chose rural areas, and some pointed out that it was the county or town where the rural hometown was located, and few people clearly went to the village. Others think it does not matter because they have to communicate with their parents, and there are more women in this group.

In the survey, in terms of employment relevance, the proportion of choosing “work in this major,” “work related to this major,” “work has nothing to do with your major,” and “flexible employment” are 7.20%, 53.50%, 23.60%, and 15.70% respectively (see Figure 12). This also shows that even agriculture related majors may not be willing to engage in work related to agriculture related majors.

#### 4.3.3. Employment Preparation and Channel Analysis

The survey shows that 47.20% of the students think it is most suitable to apply for a job one year before graduation; 38.30%, half a year before graduation; 14.20%, in the first two months. But, at the same time, 0.30% of the students are uncertain (see Figure 13). This shows that most students look forward to employment, especially in the last year of the university. They pay attention to employment and spontaneously set a timetable to guide their employment. The reason for the lower two months before graduation is that they should be busy with graduation related matters, should not be too distracted, and have no time and energy, indicating that personal arrangement is very time-based [24].

The survey shows that 77.20% of people choose to apply for jobs through job fairs and 69.60% through advertising media such as Internet and newspapers; 26.50% will apply for jobs through the talent market; 31.30% will apply for a job through relatives and friends; 15.40% will apply for jobs through independent entrepreneurship (see Figure 14).

### 4.4. The Government Establishes a Multichannel Social Support System Platform

#### 4.4.1. Creating More Jobs for Returning College Students

The level of business development is good for education. They are inextricably linked. They limit and encourage each other. First, the growth of higher education is influenced by the level of industry development. The industry, standards, and all scales of higher education define systems, models, and all scales. The supply and demand of higher education depends on the supply and demand of the market. The reaction of the development level of higher education to economic development can not be ignored. Only when the social economy develops rapidly, the total scale and speed expand, and a high-level development state is presented, can the demand for the scale and development speed of higher education expand rapidly [19]. Therefore, to solve the diligent problem of college students returning home from rural areas, the local government should find ways to promote sustained and rapid economic growth. In the relatively poor areas, especially, the government should base itself on the local reality and develop the characteristic economy according to local conditions, so that the returned college students can apply what they have learned. With the development of the economy and the expansion of the scale, the number of jobs will naturally increase. It can be seen that economic development is the fundamental measure to solve the employment problem. Only by fundamentally starting, can we completely solve the difficulties encountered by rural college students returning home for employment.

#### 4.4.2. Formulating Economic Development Policies that Give Priority to the Employment of Returned College Students

To formulate an economic development policy that gives priority to the employment of returning college students, we should first break the urban-rural dual structure and coordinate the urban-rural economic development policy. The overall planning of urban and rural economic policies does not mean that urban and rural areas should implement the same economic development policies to make the policies universal but refers to the establishment of a unified, open, and fair competitive labor market suitable for the requirements of rural industrialization and urbanization based on the existing conditions. Expand the degree of opening up, strengthen investment attraction, develop characteristic economy, people-oriented, and develop a technology intensive economy that needs scientific and technological talents.

#### 4.4.3. Encouraging College Students to Start Their Own Businesses and Expand Employment Channels

College graduates should change the traditional concept of employment. Through independent entrepreneurship, they can not only solve their own employment problems but also create more jobs for the society and solve the employment problems of more graduates. Therefore, the government should introduce relevant supporting policies. We can start from the following aspects. First, we should give certain preferential treatment to the economic entities created by college students in terms of taxation. Second, in order to ensure that college students have the start-up funds needed for entrepreneurship, the government should set up a college students' entrepreneurship guarantee fund and provide small loan guarantee for entrepreneurial college students. Moreover, the government should set up a special department to examine and approve college students' entrepreneurship projects, give policy help to college students, answer the relevant difficult problems encountered by college students, reduce the fees of relevant certificates as much as possible, and give more green lights in procedures. Finally, regularly carry out entrepreneurship service training, recommend projects within their ability to unemployed college students according to local conditions, and provide technical support and follow-up training in the later stage to help them solve their difficulties and actively guide college students to start their own businesses.

### 4.5. Supporting Measures to be Taken by Colleges and Universities

Now that the university has entered the level of interest, the quality of university graduates in the industry is gradually declining. In this environment, colleges and universities should continue to deepen the teaching modification of courses and formulate professional standards to meet the needs of the market in different situations: improving the professional competitiveness of graduates by adapting to the market, improving the curriculum, improving the quality of teaching according to each student's interests, and developing skills that are combined with unique and more talents. On the one hand, pay attention to strengthening the guidance of graduates' employment skills; on the other hand, pay attention to strengthening students' psychological counseling. Ensure that graduates have a good attitude in the process of employment and grasp the coincidence point between employment expectations and social needs.

Foreign advanced experience tells us that while colleges and universities strive to improve themselves, they are also inseparable from the support of all sectors of society. First, the government should give priority to the role of colleges and universities in promoting social and economic development, increase investment in colleges and universities, meet the funding needs of colleges and universities for scientific research projects, and improve college education programs. Only when the level of colleges and universities is improved, can they be prompted to provide higher-level educational resources for students and improve the ability of graduates to meet the needs of the labor market. Use sufficient funds to build a comprehensive employment service and build a bridge between graduates and businesspeople. Second, job companies need to build relationships with colleges and universities and allow colleges to develop professional skills that meet their needs, as their needs come from training. Avoid unnecessary friction and waste due to lack of understanding of graduates and the workplace. Not only does this help college students get good grades, but it also avoids the frustration of working in fields where skills are difficult to acquire.

### 4.6. College Students Actively Accumulate Social Capital and Pay Attention to Their Own Career Planning

#### 4.6.1. Actively Accumulating Personal Social Capital

College graduates have just left school, and their understanding of society is still in the blank stage. First, they should learn to accumulate their own social capital, start from the simplest, and start from their own side. Everyone lives in a relationship network and has their own social relations, such as relatives and friends, villagers, and classmates. These are the social capital that must be paid attention to and are the most stable social capital. These social capital will be of great help to obtain important information and good opportunities in the future.

In addition, we should pay attention to the cultivation of social skills, strengthen exchanges with people from all walks of life, and make all kinds of friends. Everyone is a part of the social network and does not exist independently. In social communication, we can not only cultivate the ability of all aspects but also expand the scope of our influence through social communication. Accordingly, we will increase our own social capital and expand the social relationship network. Due to the complex connections in the relationship network, a relatively stable network structure is formed between individuals. Due to the interaction of various actors in the structure network, social capital such as trust relationship can be generated, and the scope of this relationship network will be larger and larger, and social connections will be wider and wider. Good social capital will be of great help to graduates' employment and future career.

#### 4.6.2. Paying Attention to Their Own Career Planning

Career planning is very important for everyone. It is related to one's lifelong career path and role in society. Career planning should not start with a single interest but also consider the needs of the society and the constraints of the actual situation. Only the career planning that integrates various factors is scientific and conducive to their own development. For a newly enrolled freshman, there are many things to learn during college, but in the long run, planning their career should start from student age, which is more conducive to the pertinence of learning. Foreign universities attach great importance to the education of students' career planning. The first president of Stanford University even emphasized the importance of career planning at the opening ceremony. College is an important turning point in life. At this stage, a person gradually grows from a child to an adult with social responsibility. Most people are easy to fall into confusion at this stage, which is inevitable, but to realize their ideals and aspirations, they must quickly get out of confusion, which requires college students to formulate reasonable career planning at the beginning of enrollment. In today's social background of difficult employment, college students should formulate realistic career planning and cannot blindly follow suit. We should know how to start from the grass-roots level and not be high-profile and impetuous. This will not only help our employment but also greatly help our future development.

## 5. Conclusion

In general, from the perspective of rural entrepreneurship environment support, through empirical and typical case studies, combined with the personalized needs of college students in rural entrepreneurship, this study further clarifies the impact of entrepreneurship environment on college students' rural entrepreneurship. Solving these problems requires the joint efforts of the government, colleges and universities, students' families, and myself. On the one hand, the government and colleges and universities should introduce corresponding policies and measures to ensure the smooth employment of rural returned college students. On the other hand, college students should change their thinking, set their position according to reality, and create conditions to realize employment. Finally, family members and relatives should also take an inclusive attitude to reduce the psychological pressure of college students. With the increasingly fierce employment competition and the continuous accumulation of the number of new college students to be employed, more and more college students will choose to return home for employment. In the face of this grim prospect, all parties should make joint efforts to help rural returned college students get rid of the employment difficulties they face and realize their ideal employment.

## Figures and Tables

**Figure 1:** Rural employment and entrepreneurship process of college students.

**Figure 2:** Student origin.

**Figure 3:** Students' graduation trend.

**Figure 4:** Proportion of daily living expenses.

**Figure 5:** Proportion of economic sources.

**Figure 6:** Proportion of employment pressure sources.

**Figure 7:** College students' cognition of employment situation.

**Figure 8:** College students' views on the changes of future employment situation.

**Figure 9:** Contents that college students should improve for future employment.

**Figure 10:** Units of college students' employment intention.

**Figure 11:** Selection of employment areas for college students.

**Figure 12:** Correlation between employment and specialty.

**Figure 13:** Cognition of employment preparation period.

**Figure 14:** Selection of employment channels.

**Table 1:** Calculation steps of factor analysis method.

Sample variable	*X*_1_	*X*_2_	...	*X*_*P*_
1	*X*_11_	*X*_12_	...	*X*_1*P*_
2	*X*_21_	*X*_22_	...	*X*_2*P*_
...	...	...	...	...
*n*	*X*_*n*1_	*X*_*n*2_	...	*X*_*nP*_

## Data Availability

The labeled dataset used to support the findings of this study is available from the author upon request.
